The article "The Molecular Mechanisms of Defective Copper Metabolism in Diabetic Cardiomyopathy" was published in 2022. Journal: Oxid Med Cell Longev.

# The Molecular Mechanisms of Defective Copper Metabolism in Diabetic Cardiomyopathy

**DOI:** 10.1155/2022/5418376

**Published:** 2022-10-04

**Authors:** Xiangning Cui, Yan Wang, Han Liu, Mengjun Shi, Jingwu Wang, Yifei Wang

**Affiliations:** ^1^Department of Cardiovascular, Guang'anmen Hospital, China Academy of Chinese Medical Sciences, Beijing 100053, China; ^2^First Clinical Medical School, Shandong University of Traditional Chinese Medicine, Jinan, Shandong 250000, China; ^3^Affiliated Hospital of Shandong University of Traditional Chinese Medicine, Jinan, 250000 Shandong, China

## Abstract

Copper is an essential trace metal element that significantly affects human physiology and pathology by regulating various important biological processes, including mitochondrial oxidative phosphorylation, connective tissue crosslinking, and antioxidant defense. Copper level has been proved to be closely related to the morbidity and mortality of cardiovascular diseases such as atherosclerosis, heart failure, and diabetic cardiomyopathy (DCM). Copper deficiency can induce cardiac hypertrophy and aggravate cardiomyopathy, while copper excess can mediate various types of cell death, such as autophagy, apoptosis, cuproptosis, pyroptosis, and cardiac hypertrophy and fibrosis. Both copper excess and copper deficiency lead to redox imbalance, activate inflammatory response, and aggravate diabetic cardiomyopathy. This defective copper metabolism suggests a specific metabolic pattern of copper in diabetes and a specific role in the pathogenesis and progression of DCM. This review is aimed at providing a timely summary of the effects of defective copper homeostasis on DCM and discussing potential underlying molecular mechanisms.

## 1. Introduction

Diabetic cardiomyopathy (DCM) is one of the major complications of type 1 and type 2 diabetes [1, 2], accompanied by altered cardiac energetics, impaired mitochondrial function, and oxidative stress, manifested as heart failure in the absence of coronary artery disease, hypertension, and valvular heart disease [1, 3–6]. So far, the mechanism is not clear, and there is no direct and effective treatment for DCM [1, 7, 8]. Studies have shown that copper regulation defects are related to the pathogenesis of DCM [9–11]. Copper is an essential trace element in human body. It exists in reduced form (Cu^+^) in cells and in higher oxidation state (Cu^2+^) in extracellular [12, 13]. Copper ions are widely distributed in human muscle, bone, liver, and blood and participate in biological processes such as energy metabolism, electrolyte balance, cell apoptosis and autophagy [14], and protein redox [13].

It has been demonstrated in animals and humans that, regardless of the presence or severity of diabetic complications, diabetic patients have higher levels of copper in plasma and urine compared with nondiabetic controls [10, 15, 16]. Imbalance between intracellular and extracellular copper pools may elevate plasma copper in diabetes and decrease copper content in cardiomyocytes [17–19]. And consistent with that increases in circulating copper concentrations and 2~3-fold increases in extracellular myocardial Cu^2+^levels, but decreases in intracellular myocardial Cu^+^ levels, were reported in humans and rodents with DCM [18]. The reduced myocardial copper content and elevated systemic and total cardiac copper content in DCM reflect defective excretion and uptake of copper [10, 20, 21]. Differ from those in Wilson's disease which is caused by mutations in copper-transporting ATPase (ATP7B) [22], the copper metabolism defect in diabetes leads to a significant increase in the level of copper in blood and a decrease in the content of copper in the liver [23], resulting in changes in the processing of copper in the liver and a decrease in the clearance rate of copper in circulation.

The article "The Molecular Mechanisms of Defective Copper Metabolism in Diabetic Cardiomyopathy" was published in 2022. Journal: Oxid Med Cell Longev.

Copper deficiency in myocardial cells can lead to impairment of energy use by the heart, reduced ability of the heart to contract, and induce cardiomyopathy [24], while high levels of Cu have been positively correlated with reactive oxygen species (ROS) generation [16]. At the same time, accumulation of catalytically active Cu^2+^ in the cardiac extracellular myocardial induces copper toxicity, which is proposed as an important catalyst of cardiovascular damage in diabetes [11, 17]. Copper toxicity leads to protein oxidation, glutathione (GSH) depletion, lipid damage, and redox imbalance [13, 25], which could cause acute impairment of cardiac function, exacerbating chronic underlying damage. Therefore, copper metabolism defect is closely related to the pathogenesis of DCM, which is expected to become another unique angle to explore the pathogenesis of DCM.

## 2. Copper-Relating Proteins and Pathological Processes in DCM

In physiological state, copper ions are absorbed through diet and reduced to Cu^+^ under the action of cell surface reductase in the small intestine and then absorbed by copper transporter 1 (CTR1) into cells to realize the transmembrane transport of copper ions [26]. Once inside the cell, free copper ions are immediately isolated by chaperone proteins and then transported to copper enzymes in the different cytosolic compartment by metal ligands (ATOX1, CCS) or alternative ligands (CuL, GSH) [27]. In the liver, it is oxidized by ceruloplasmin (CP) [28] and binds with related proteins, which is released into the blood and transported to relevant tissues and organs to participate in the regulation of life processes [13, 29] (Figure 1).

The article "The Molecular Mechanisms of Defective Copper Metabolism in Diabetic Cardiomyopathy" was published in 2022. Journal: Oxid Med Cell Longev.

The activity of the copper transporters and Cu-transporting ATPases [18] is implicated in DCM, regulating mitochondrial respiration, antioxidant defense, iron metabolism, and connective tissue crosslinking [33]. The functions of copper heavily rely on intact mitochondrial respiration [34–37]. The regulatory mechanisms of copper are complex, involving a range of signal transduction and molecular and metabolic pathways. Therefore, we summarized the physiological role of related copper chaperone protein and its mediated cardiac disease (Table 1), as well as the role of copper chaperones and copper transporters in pathological processes in DCM.

### 2.1. Copper Chaperones and Pathological Processes in DCM

#### 2.1.1. CCO

Copper-dependent CCO is the mitochondrial respiratory chain complex IV, which contains copper and heme as required cofactors in mitochondria-encoded DNA subunits (I, II, and III), playing a critical role in oxidative phosphorylation as the catalytic core of the oxidase complex. Several copper chaperones deliver copper to CCO, including CCO copper chaperone 11 (COX11), COX17, COX19, and COX23 and synthesis of CCO 1 (SCO1) and SCO2. Therefore, when CCO activity decreases, mitochondrial function is inhibited. Some early studies found that copper deficiency can reduce CCO activity in the heart [35–37, 55]. Thus, copper deficiency in cardiomyocytes significantly reduces the expression of copper chaperones and enzymatic activity of CCO, halving the level of copper in the left ventricle and decreasing the systolic function of the left ventricle in DCM [9].

#### 2.1.2. The SOD Family

The SOD family, another copper transporter, including SOD1, SOD2, and SOD3, promotes the progression of DCM to heart failure disease through oxidative stress pathway. Copper zinc superoxide dismutase (SOD1) is a critical enzyme against ROS by catalyzing dismutation of the deleterious superoxide radical (O^2-^) to molecular oxygen or hydrogen peroxide, which is in turn reduced to water by other [56]. Cytosolic SOD1 transmit signals from oxygen and glucose to affect respiration rates via an interaction with casein kinase 1-*γ* [57]. SOD1 also is required for prevent protein misfolding, aggregation, and inactivation after copper enters mitochondria [58], for which delivery of copper to SOD1 by the Cu-CCS complex permits formation of disulfide bonds in SOD1 [58]. The latest findings that high-fat decreased the levels of copper chaperone for SOD1 (CCS) in cells, which decreased the activity of SOD1 and antioxidant capacity, manifested as an increase in ROS in the vivo [59]. Moreover, diabetic rats had low SOD1 activity that was reduced even further when diabetic rats were fed with low-copper diets [60].

The article "The Molecular Mechanisms of Defective Copper Metabolism in Diabetic Cardiomyopathy" was published in 2022. Journal: Oxid Med Cell Longev.

Therefore, SOD1 activity was significantly inhibited in the presence of copper deficiency in DCM. In the high-fat and high-sugar environment of DCM, the downregulation of SOD1 activity may lead to the destruction of mitochondrial biological functions, such as abnormal biological activity of mitochondrial proteins, the decreased ability of scavenging free radicals, decreased mitochondrial respiration rate, and increased ROS level. In DCM, although the body is in a high glucose state, the glycolysis metabolism is impaired and cardiomyocytes rely on mitochondrial oxidized fatty acids as the main energy source [61]. When mitochondrial function is impaired, oxidative utilization of fatty acids in cardiomyocytes is reduced, resulting in excessive accumulation of free fatty acids, which aggravates lipotoxic injury.

Manganese-containing SOD2 (MnSOD) localizes to mitochondria and serves as the first line of defense against mitochondrial respiration-generated oxidative stress. Although SOD2 does not bind to copper, it indirectly regulates the activity of copper-containing SOD1. SOD2-deficient mice show increased release of superoxide anion radical derivatives and impaired SOD1 activity, which causes heart failure (HF) [45]. These mice exhibit myocardial damage, with enlarged mitochondria, loss of cristae, and fewer myofilaments, as well as lipid peroxidation and activation of apoptosis. In addition, NAD^+^ redox imbalance promoted SOD2 acetylation, protein oxidation, and impaired energetics in DCM [62].

Copper-bound SOD3, which is primarily expressed in blood vessels and is extracellularly localized, has also been linked to heart disease. Activity and/or expression of copper-bound SOD3 was reported to be decreased in animal models and humans with hypertension, HF, and coronary heart disease [63–65], decreasing the antioxidant capacity of the body. SOD3 can catalyze the dismutation of superoxide radical to hydrogen peroxide and molecular oxygen, protecting the heart from oxidant-induced fibrosis, apoptosis, and loss of function [47]. As a sensitive indicator of copper status [66], serum SOD3 activity decreased in DCM [67], and the reduction of its antioxidant defense ability aggravated the toxic damage caused by Cu^2+^.

#### 2.1.3. MT

MTs are cysteine-rich, low molecular weight proteins that bind to copper and serve as intracellular copper scavengers. Liver and kidney MT and plasma CP levels were elevated in diabetic rats [60], suggesting that there may be elevated intracellular copper levels in the liver and kidney in diabetes mellitus. When cytosolic copper reaches excess, it is bound by MT, then ATP7A relocalizes to the plasma membrane where it acts as a copper exporter, thus achieving intracellular copper equilibrium.

The article "The Molecular Mechanisms of Defective Copper Metabolism in Diabetic Cardiomyopathy" was published in 2022. Journal: Oxid Med Cell Longev.

The formation of copper-thiolate clusters in MTs sequesters excess copper in cells and thereby minimizes copper toxicity [68]. In addition to isolating excess copper, T also has a variety of regulatory effects in DCM. It has been confirmed that MT can modulate various stress-induced signaling pathways such as Wnt, NF-*κ*B, and PI3K, to alleviate diabetes and diabetic complications [69]. MT prevents DCM by inhibiting ROS production [70], attenuating oxidative stress, and increasing expression of proteins associated with glucose metabolism [71] as well as suppressing NOX-dependent nitrosative damage and cell death [72].

#### 2.1.4. LOX

The copper-dependent LOX enzyme is critical to catalyze lysine-derived crosslinking of collagen and elastin fibrils in the extracellular matrix [73]. Myocardial fibrosis, mostly characterized by the excessive interstitial and perivascular deposition of collagen types I and III fibers [74], is a biological process involving inflammatory response and reactive ROS accumulation leading to fibroblast activation [75].

LOX-mediated cross-linking of collagen types I and III fibrils leads to the formation of stiff collagen types I and III fibers, as well as their subsequent tissue deposition in patients with enhanced myocardial stiffness and HF [76–78]. It is thus conceivable that when Cu^2+^ increases, LOX is activated and its expression is up-regulated, which accelerates the process of collagen fiber cross-linking and promotes myocardial fibrosis [79]. Inhibition of collagen and elastin crosslinking reduces the tensile strength and elastic properties of connective tissues, which results in a failure to maintain normal cardiac contraction and the development of concentric cardiac hypertrophy [53, 54].

#### 2.1.5. Glutathione (GSH)

Glutathione acts as a copper chaperone to protect cells from copper toxicity, and in turn, excessive copper also destroys glutathione levels [80]. In malnutrition [81], cell differentiation [82], even aging cells [83], or a certain stage of development, the overall content of glutathione will be hit a second time, aggravating the toxic damage of copper, thus triggering or worsening the ongoing body lesions, such as DCM [18], heart failure [84], and cancer [85].

### 2.2. Copper Transporters and Pathology in DCM

#### 2.2.1. CTR

CTR1 is the only known plasma membrane copper importer with high affinity in mammalian cells so far that localizes to the plasma membrane and endosomes [86, 87], whereas CTR2 is a low-affinity copper importer that localizes to endosomes and lysosomes. Ablation of CTR2 reduces the generation of truncated CTR1 lacking a copper-binding echo domain and, thus, increases tissue copper contents [88]. Its abundance and location determine the rate of copper import [89] and regulate the redox state of Cu^+^ [90], playing an important role in regulating intracellular copper homeostasis and copper bioavailability. In the presence of excess copper, CTR1 can be internalized from the plasma membrane into the endocytic body [90] to protect cells from copper poisoning. Endosomal CTR1 can then be degraded by the proteasome or recycled back to the plasma membrane [91]. However, the localization of CTR1 in polarized epithelial cells has been controversial [92, 93], leading to doubts about the universality of this regulatory mechanism.

The article "The Molecular Mechanisms of Defective Copper Metabolism in Diabetic Cardiomyopathy" was published in 2022. Journal: Oxid Med Cell Longev.

A copper-deficient diet reduces heart CTR2 protein expression by 46% compared with a copper-adequate diet in rats, demonstrating a potential association of a reduction in CTR2 in cardiac copper deficiency and heart disease [94]. However, the specific mechanism remains unclear and needs further study. Unlike the hypertrophy of myocardium caused by insufficient copper levels throughout the body in the pressure load type, copper levels in the DCM are high in the blood throughout the body but low in the myocardium cells [18] that may be related to the deficiency of copper uptake by cells due to the decreased expression activity of CTR1. Just as Zhang et al. reported that the expression of the CTR1 gene was downregulated in hearts of rats with DM, which is consistent with impaired cardiac copper uptake in DM [18]. Therefore, the activity and expression of CTR1 play a key role in copper metabolism defects and cardiac hypertrophy in DCM.

#### 2.2.2. ATP7A and ATP7B

ATP7A and ATP7B are copper exporters belonging to the P-type ATPase family and contain an ATP hydrolysis domain to provide energy for copper trafficking. ATP7A is ubiquitously expressed, with the exception of the liver in normal states. In specific cell types, ATP7B replaces ATP7A and relocates to vesicles to facilitate their excretion through bile [95, 96]. When cytosolic copper level rises, ATP7A or ATP7B traffics to the plasma membrane, pumping excess copper into the extracellular space, or into bile in the case of the liver, to reduce the intracellular copper level [97]. By contrast, when the intracellular copper level is low, ATP7A or ATP7B recycles to TGN and transports copper from the cytoplasm into the Golgi. Genetic studies have shown that copper export is the main way to reduce copper toxicity, because ATP7A-deficient cells are much more sensitive to excessive copper than lack MT [98].

The article "The Molecular Mechanisms of Defective Copper Metabolism in Diabetic Cardiomyopathy" was published in 2022. Journal: Oxid Med Cell Longev.

#### 2.2.3. CP

CP carries more than 90% copper in plasma that is critical for maintaining activities of copper-dependent enzymes, including SOD1 and SOD3, and thus the removal of oxygen radicals [99]. Hyperglycemia may increase free Cu^2+^ in the extracellular space by impairing the Cu-binding properties of ceruloplasmin and albumin, possibly via nonenzymatic glycation [100–102], causing increased levels of Cu^2+^ bound at molecular sites other than those in physiological Cu proteins, so that it is catalytically active. CP also is an oxidase for NO that converts NO to nitrite in vivo [103, 104]. Circulating CP is negatively associated with NO bioavailability, presumably due to increased conversions of NO, and enhanced oxidative stress which in turn adversely impacts heart function [105].

CP can be used as a redox marker of heart failure severity [106]. Previous studies have shown that increased levels of CP are associated with increased risk of developing heart failure. Serum CP levels are significantly raised in patients with diabetes [107] that exacerbates the progression of DCM to heart failure. CP is an independent predictor of all-cause mortality in patients with heart failure [108], but the specific pathogenesis is still unclear.

## 3. Defective Copper Metabolism and DCM

DCM is characterized by myocardial remodeling, including cell death, myocardial fibrosis, and hypertrophy, leading to diastolic dysfunction with or without systolic dysfunction. It has been reported that changes in endothelial cells [109] and cardiomyocytes [110] caused by diabetes are one of the main reasons for the occurrence and development of DCM. Biopsy showed that the apoptosis of a diabetic heart was 85 times higher than that of the nondiabetic heart, indicating that cardiomyocytes in diabetes were sensitive to suffer cell death [111]. Essentially, cell death is considered to be the terminal pathway of DCM cardiomyocytes [112].

Defective copper metabolism produces cytotoxicity, also known as copper toxicity, that damages mitochondrial structure and function [45], lipid metabolism, cellular autophagy, and cell death through excessive oxidative stress and inflammatory response [113–116]. As the contractile unit of myocardial tissue, myocardial cells' apoptosis triggers a series of reactions such as cell hypertrophy and fibrosis, leading to myocardial diastolic and contractile dysfunction and exacerbating heart failure [117–119]. Altered myocardial copper-trafficking is a key pathogenic process in diabetes-evoked heart failure [9]. Therefore, this chapter mainly introduces the influence of copper metabolism deficiency on DCM from three aspects: cell death, myocardial hypertrophy, and myocardial fibrosis.

The article "The Molecular Mechanisms of Defective Copper Metabolism in Diabetic Cardiomyopathy" was published in 2022. Journal: Oxid Med Cell Longev.

### 3.1. Cell Death

Apoptosis and mitochondrial autophagy are common phenomena in the occurrence and development of diabetic cardiomyopathy [112]. Copper can induce multiple forms of cell death (Figure 2), including apoptosis and autophagy, through various mechanisms, including reactive oxygen species accumulation, proteasome inhibition, and antiangiogenesis [120].

#### 3.1.1. Autophagy

Elevated copper in senescent mouse embryonic fibroblasts (MEF) was accompanied by elevated levels of high-affinity CTR1, diminished levels of ATP7A, and enhanced antioxidant defense reflected by elevated levels of GSH, SOD1, and glutaredoxin 1 (Grx1) [126]. Mitochondria is sensitive to changes in the environment in the cell, and the internal environment of the upheaval caused the change of mitochondrial membrane potential and the integrity of the structure damage. Recent studies have found that the chelation of autophagosomes to relevant targets has high specificity, which is the main way to selectively remove abnormal mitochondria. The lysosomal degradation of damaged mitochondria, called mitophagy, is an important cellular self-protective. Autophagy is a process that removes abnormal proteins and organelles [127] and maintains cell homeostasis by removing misfolded proteins and damaged organelles and invading microorganisms through lysosomes [128]. Autophagy plays an important role in cellular copper clearance. The means by which the copper metabolism and autophagy pathways interact mechanistically is vastly unexplored.

Metabolomics analysis reveals that metabolites were overall downregulated in cardiomyocytes after copper treatment [129], with a principal impact on the metabolic pathways including glycerophospholipid metabolism, fatty acid elongation, and fatty acid degradation, which were related to autophagy. Copper can mediate increased autophagy and metabolic pathway disturbance to induce myocardial injury. Copper is required for the activity of the autophagic kinases ULK1 and ULK2 (ULK1/2) through a direct Cu-ULK1/2 interaction [130]. Genetic loss of the copper transporter CTR1 or mutations in ULK1 that disrupt the binding of copper reduced ULK1/2-dependent signaling and the formation of autophagosome complexes. Increased levels of intracellular copper are associated with starvation-induced autophagy and are sufficient to enhance ULK1 kinase activity and, in turn, autophagic flux [130]. Activation of autophagy, observed in liver tissues from patients with Wilson disease and from ATP7B-deficient animals, protects hepatocytes from copper-induced apoptosis [131]. ATP7B contains a number of potential binding sites for LC3, a central protein in the autophagy pathway, the so-called LC3 interaction regions (LIRs) [132]. The conserved LIR3, located at the C-terminal end of ATP7B, was found to directly interact with LC3B in vitro [132].

The article "The Molecular Mechanisms of Defective Copper Metabolism in Diabetic Cardiomyopathy" was published in 2022. Journal: Oxid Med Cell Longev.

MTOR is a protein kinase that negatively regulates autophagy. Excess copper inhibited the activity of mTOR through suppressing mRNA and protein expressions in mTOR, which in turn upregulated expression levels of ULK1 and initiated autophagy [122]. The toxic effects of copper induced a clear impairment of autophagy [133], through the absence of phagosomes and the significant downregulation mRNA transcript levels of microtubule-associated protein LC3, which is often associated to an increase of apoptotic activation. Simultaneously, copper ion could inhibit the activity of ATG4B that plays a vital role in autophagy process via undertaking priming and delipidation of LC3, followed by autophagy suppression [134]. Autophagy has been linked to Cu-induced toxicity. Loss of LC3B resulted in aggravated lung injury induced by copper oxide nanoparticles (CuONPs) [135], which was probably due to the blockade of mitophagy and consequently the accumulation of aberrant mitochondria with overloaded copper ions. CuSO4 induced autophagy through Akt/AMPK/mTOR pathway and significantly induced the production of mitochondrial reactive oxygen species (mtROS) [136]. MtROS is the original cause in CuSO4-induced apoptosis and autophagy [136]. After copper accumulation, it activates excessive autophagy, disturbs mitochondrial dynamics, and aggravates REDOX imbalance, forming a vicious cycle [137].

#### 3.1.2. Cuproptosis

In mitochondria, excessive copper directly binds to lipoylated components of TCA that results in aggregation of lipoylated protein and subsequent iron-sulfur cluster protein loss, leading to proteotoxic stress and ultimately cell death, also known as cuproptosis [113, 115]. Unlike known mechanisms of cell death, such as apoptosis [138], necroptosis [139], pyroptosis [140], and ferroptosis [141], cuproptosis does not involve either the cleavage or activation of caspase 3 activity, the hallmark of apoptosis [113, 142], which is a mechanism distinct from known cell death pathways.

FDX1 and protein lipoylation are the key regulators of copper ionophore–induced cell death [113]. Elesclomol, as one of the common copper ion carriers, is an effective tool to study copper toxicity [143]. Elesclomol directly binds to the mitochondrial reductase FDX1, resulting in the biosynthesis of Fe-S clusters inhibited [116]. Fe-S cluster–dependent processes include the energy transformation and metabolite conversion via mitochondrial respiration (complexes I–III), the TCA cycle, and numerous anabolic and catabolic reactions [144]. As is common for mitochondrial disorders, the clinical phenotypes of Fe-S diseases are associated with respiratory deficiencies and severe metabolic dysfunctions [145, 146]. Elesclomol-Cu^2+^ complex, as a new substrate for FDX1 reduction [116], reduces Cu^2+^ in mitochondria to Cu^+^ to promote the production of higher levels of ROS, ultimately leading to cell death [147–150]. FDX1 activity and increased mitochondrial-dependent energy metabolism are strong inducers of the cytotoxic effects of elesclomol-mediated cuproptosis [116]. In addition, cuproptosis caused by depletion of intracellular natural copper companion GSH is associated with decreased lipoylation and increased DLAT oligomerization [113].

The article "The Molecular Mechanisms of Defective Copper Metabolism in Diabetic Cardiomyopathy" was published in 2022. Journal: Oxid Med Cell Longev.

Cuproptosis, as a mechanism proposed in the latest studies, mainly focuses on the intervention of cancer treatment [113, 115]. It is a new research hotspot to kill cancer cells [120] by targeting excessive copper delivery to cancer cells to destroy mitochondrial respiration and cut off energy supply, thus mediating cancer cell death. Current studies show that the effects of excessive copper on the heart mainly focus on oxidative stress or inflammation-mediated cell death, but there is no relevant study on the mechanism of cuproptosis. It is known that in DCM, there is an excess of copper in systemic plasma and a deficiency in cardiomyocytes and that coronary capillaries in the heart penetrate deep into myocardial tissue to provide energy to the myocardium, while cuproptosis often occurs in cells with high energy metabolism, such as rich mitochondria. Therefore, we can speculate that the excess copper in plasma may damage mitochondria in vascular endothelial cells through cuproptosis or oxidative stress pathway and then affect the function of cardiomyocytes. Of course, further experimental studies are needed to confirm this idea. However, cuproptosis may provide a new direction for the pathological change mechanism of DCM.

#### 3.1.3. Pyroptosis

In various diseases, including diabetes, due to the lack of a resolution phase of the inflammatory state, myocardial inflammation contributes to pathological hypertrophic growth and leukocyte-mediated death of cardiomyocytes [151]. Inflammasome stimulation is a two-step process requiring priming by inflammatory stimuli. The first step is NF-*κ*B transcriptional upregulation of NLRP3 and pro-IL-1*β*. The second step involves DAMP-mediated inflammasome assembly, causing oxidative stress and inflammation-induced programmed cell death, also known as pyroptosis [124].

The article "The Molecular Mechanisms of Defective Copper Metabolism in Diabetic Cardiomyopathy" was published in 2022. Journal: Oxid Med Cell Longev.

Inflammasome expression is markedly increased in rodent diabetic hearts via oxidative stress-dependent thioredoxin-interacting/inhibiting protein (TXNIP) activation, showing elevated caspase-1 and IL-1*β* activation [152]. Moreover, excessive cytokines, in turn, exacerbate mitochondrial dysfunction in a positive feedback loop [153, 154]. In diabetes, mitochondrial damage has been detected as an important contributor to inflammasome assembly through the release of mitochondrial DNA and ROS. Excess Cu induced pyroptosis by generating ROS in hepatocytes, and the inhibition of Caspase-1-dependent pyroptosis might attenuate Cu-induced apoptosis [155]. In addition, there are research findings that ER stress also participated in regulating Cu-induced pyroptosis in jejunal epithelial cells via the IRE1*α*-XBP1 pathway [156], which provided a novel view into the toxicology of copper.

#### 3.1.4. Apoptosis

Apoptosis, also known as programmed cell death, is a modulated, noninflammatory cell death pathway. The different apoptosis pathways are triggered by copper at different time points of the exposure period, as the increase in transcripts was sequential [121], instead of simultaneous. The higher incidence of TUNEL-positive cells, in gill epithelia of the exposed fish, proved that copper induced apoptosis [121]. Recent animal experiments indicated that the copper exposure promotes apoptosis and autophagy through oxidative stress in pig testicular [157] and rat kidneys [158]. In humans, copper can also induce apoptosis and autophagy through oxidative stress-mediated mitochondrial dysfunction in male germ cells [159].

Apoptosis seems to be initiated via intrinsic pathway (caspase-9), through p53 activation and then followed by the extrinsic pathway (caspase-8) and finally by the caspase-independent pathway (AIF) [121]. Furthermore, excessive copper not only can destroy the stability of iron-sulfur clusters [113, 160] but also enhance the production of extremely destructive free radicals [114, 161]. Disruption of the superoxide anions-mitophagy regulation axis mediates copper oxide nanoparticle-induced vascular endothelial cell death [162]. Another study showed that copper oxide nanoparticles can induce oxidative DNA damage and cell death via copper ion-mediated P38 MAPK activation in vascular endothelial cells [163]. The mitochondrial membrane potential decreased, while the number of apoptotic cells increased, as a result of oxidative stress [157].

Nishikawa et al.'s group provided strong evidence that under hyperglycemic conditions, ROS in vascular endothelial cells are derived from the mitochondrial ETC, as evidenced by an inhibition of increased ROS production by treatment with an uncoupling agent or a complex II inhibitor [164]. Elevated catalytically active Cu^2+^ in the extracellular myocardial could overwhelm antioxidant defenses, such as those catalyzed by extracellular SOD3 [165], causing enhanced ROS production through Fenton or Haber-Weiss chemistry, thus elevating oxidative stress [10, 19, 166]. ROS have been proposed to contribute to fibrosis, ventricular remodeling, or direct damage to cardiomyocyte [70]. However, given that direct comparison of cytosolic versus mitochondrial sources of ROS production in the diabetic heart are limited, it is difficult to evaluate the relative contributions of each ROS-producing enzyme.

The article "The Molecular Mechanisms of Defective Copper Metabolism in Diabetic Cardiomyopathy" was published in 2022. Journal: Oxid Med Cell Longev.

### 3.2. Cardiac Hypertrophy

Copper deficiency causes cardiac hypertrophy by impairing mitochondrial function and energy production, evidenced by increases in mitochondrial compensatory biogenesis and size and mitochondrial ultrastructural deteriorations, as well as a decrease in the number or loss of cristae [167, 168]. Consistently, Oster et al. showed that cardiac copper levels positively correlated with the cardiac ejection fraction in 27 patients with coronary heart disease who underwent coronary artery bypass surgery [169]. Copper deficiency resulted in increases in the size and reduction in the number of cardiomyocytes in the heart. A study suggests that a direct reduction in the size of some hypertrophic cardiomyocytes and a replication of other hypertrophic cardiomyocytes with reduced size make a significant contribution to the regression of copper-deficient heart hypertrophy, leading to normalization of the size and the number of cardiomyocytes in the heart [170]. Early studies have found that copper deficiency can lead to increased mitochondrial volume density, crest disorder, nonaligned myofibrils with disturbances at Z-bands in cardiomyocytes [171]. Additionally, all copper-depleted rats demonstrated fragmented basal laminae at capillary-myocyte interface. Increased QRS amplitude and notching and greater QT intervals were displayed. These results suggest that capillary-myocyte interface changes may play an important role in the developing pathology of copper depletion.

Decreases in the delta subunit protein and beta mRNA transcript have been reported for ATP synthase as a function of copper deficiency. Oxidative phosphorylation appears to occur unaltered in the copper-deficient state, but the limited data available suggest that copper, either indirectly or directly, alters ATP synthase function [172]. When glycolysis is inhibited and ATP production cannot meet the energy requirements of the cell, that activates AMPK and increases the oxidation requirements of fatty acids rather than fat production [173]. The lipid environment has a significant steric effect on the Cu^2+^ binding conformation that Cu^2+^ binding to lipid membrane surfaces lead to lipid oxidation [174]. However, higher copper levels did not contribute to fatty acid oxidation and fat decomposition. A repeated measurement study shows that high copper exposure may elevate blood lipid levels as well as disturb processes related to oxidative stress and inflammation responses [175]. This phenomenon is not only reflected in adults but also in children. Children with higher plasma levels of copper tended to have a higher regional and overall body fat deposition [176].

The article "The Molecular Mechanisms of Defective Copper Metabolism in Diabetic Cardiomyopathy" was published in 2022. Journal: Oxid Med Cell Longev.

The shift in cellular metabolism from glycolysis to oxidative phosphorylation may promote protein toxicity [116]. Changes in cell metabolism can affect the cell's ability to inhibit proteasome function, and disturbances in proteasome function can lead to changes in cell energy metabolism. The feedback loop may result from the energy requirements of protein synthesis [177] and decomposition [178], as well as the recovery of amino acids produced by damaged, oxidized, and dysfunctional proteins [179], which are the building blocks of protein synthesis, metabolism, and redox pathways [180, 181]. In conclusion, both copper deficiency and excessive copper can induce cardiac hypertrophy, which can lead to redox imbalance through its effects on mitochondrial respiration, protein metabolism, and lipid metabolism, and eventually induce cell hypertrophy or loss.

### 3.3. Myocardial Fibrosis

The ratio of type III/type I collagen had significantly increased [182] of rat heart in copper deficiency-induced cardiac hypertrophy. In hearts of rats with DM, increased extracellular Cu^2+^ increases gene expression of TGF-*β*, Smad4, and collagens, which results in collagen deposition and increases the formation of AGEs of collagens [166]. The advanced glycation end products (AGEs), whose production is enhanced in diabetes, can forge cross-links between long-lived fibrous proteins [183] and act as localized endogenous chelators to increase tissue-Cu binding in extracellular matrix [184–186]. Cu^2+^ thus demonstrated can be designated as “chelatable” and is considered as a surrogate measure for catalytically active “free” Cu^2+^. Cu^2+^ bound to pathogenic sites, such as those in AGE-modified proteins [185], is thought to undergo instantaneous reduction to Cu^+^ by reducing agents in the extracellular fluid, such as ascorbate ions, triggering reactions with ROS [19, 187, 188]. Besides, inflammatory cytokines also activate cardiac fibroblasts, inducing excessive interstitial fibrosis formation, leading to cardiac dysfunction [189].

The article "The Molecular Mechanisms of Defective Copper Metabolism in Diabetic Cardiomyopathy" was published in 2022. Journal: Oxid Med Cell Longev.

Heart failure in diabetes may thus be explained in part by defective distribution of the two copper valence states and the myocardial damage that ensues [190]. A meta-analysis including 1504 subjects indicated that serum copper levels were significantly increased in patients with heart failure [191]. It identified a significant association between high serum copper and HF which was further confirmed in another experimental observational study. Serum copper was increased both in acute and chronic heart failure [192] and correlated with LV systolic and diastolic function [193, 194], also correlating with higher one-year mortality and morbidity [192].

## 4. Interventions for Cuproptosis Associated with DCM

Many studies have shown that cardiac hypertrophy caused by pressure overload can be promoted by supplementing copper to promote the regression of cardiac hypertrophy [195–197]. However, for patients with diabetes and DCM, copper deficiency in cardiomyocytes is not due to insufficient dietary intake, but the inability of excess copper ions in blood to enter cells. Therefore, regulation of copper chaperone and transporter bioactivity may be an effective target for regulating the intracellular and intracellular balance of copper ions in DCM, on the one hand, promoting the uptake of copper ions required by cardiomyocytes to maintain normal cellular respiration and, on the other hand, promoting the excretion of excess copper ions from plasma to reduce copper toxic damage.

Triethylenetetramine (also known as trientine, or TETA) is approved for the treatment of Wilson's disease [198] that also is employed as an experimental therapeutic molecule in diabetes where it improves cardiac structure in patients with DCM [199] and left ventricular hypertrophy [200]. TETA can prevent excessive cardiac collagen deposition, improve cardiac structure and function, and restore antioxidant defense by promoting copper excretion [196]. Consequently, it is now undergoing phase II clinical trials to assess its safety and efficacy as a therapy for heart failure in diabetes [20]. However, direct in vivo evidence that TETA can improve cardiac function in heart failure has hitherto been lacking. More recently, study confirmed that it also induces autophagy and reduces weight gain in mice fed a high-fat diet (HFD) by the activation of an AcCoA-depleting enzyme [201], thus making it a candidate pharmacotherapeutic for the cardiovascular complications of diabetes.

TETA is metabolized by acetylation and has been found in plasma and urine of healthy and diabetic patients treated with TETA [202], and they may play a role in TETA-mediated copper chelation and restoration of physiological copper regulation in diabetic patients. The uptake of Cu^2+^-TETA by cardiomyocytes was ATP-dependent. It is thus concluded that the formation of Cu^2+^-TETA facilitates copper accumulation in cardiomyocytes through an active CTR1-independent transportation process [203]. Low-dose TETA functions as a copper chaperone, selectively delivering copper to the copper-deprived heart through an active transportation; in higher doses, TETA simply retains its chelator function, removing copper from the body by urinary excretion [196]. Although the highly selective Cu^2+^ chelator TETA efficiently treats DCM, long-term clinical studies are necessary to determine whether the improvement of cardiac function by TETA is associated with long-term benefits for mortality.

The article "The Molecular Mechanisms of Defective Copper Metabolism in Diabetic Cardiomyopathy" was published in 2022. Journal: Oxid Med Cell Longev.

Long-term use of copper binding compounds including copper ionophores will disturb the homeostasis of base metals and cause serious side effects. Lack of selectivity is a major challenge in this field, and novel copper-binding compounds that selectively target cancer cells are highly sought after. New disulfiram derivatives, an FDA-approved drug to treat chronic alcoholism, as monoacylglycerol lipase-selective inhibitors [204] and aldehyde dehydrogenase1a1-selective inhibitors [205], are beneficial for the treatment of a wide range of diseases, such as inflammation [206, 207], metabolic disorders [208], and cancer [209]. Disulfiram treatments augmented hepatic copper in mice, markedly moderated body weight, and abolished the deleterious systemic changes associated with a high-fat diet [210]. Disulfiram specifically altered systemic copper in mice and altered hepatic copper metabolism, perturbing the incorporation of copper into ceruloplasmin and subsequently reducing serum copper concentrations [211, 212]. Serum ceruloplasmin represents a biomarker for disulfiram activity. These results indicate that copper ion carrier can not only reduce the high copper level in DCM and improve copper metabolism defects but also have a potential therapeutic effect on obesity caused by lipid metabolism disorder [211]. Moreover, recent studies have shown that cell lines with high levels of lipoylated proteins are sensitive to copper-induced cell death, suggesting that cupric treatment should target diseases with this metabolic signature [113]. Future clinical trials of copper ionophores using a biomarker-driven approach should therefore be considered.

## 5. Conclusions and Perspectives

Studies on copper metabolism defects in DCM have attracted extensive attention. Copper metabolism disorder leads to copper deficiency in cardiomyocytes and excessive copper in plasma, which will damage cardiac structure and function to varying degrees in DCM. Copper deficiency mainly mediates cardiac hypertrophy and induces or aggravates cardiomyopathy. Copper excess mediates many types of cell death, including apoptosis, autophagy, pyroptosis, and, more recently, cuproptosis, which also induces and aggravates myocardial fibrosis. Redox imbalance and inflammatory response play an important role in bridging these lesions, linking various mechanisms inside and outside the cell. In addition to heart damage caused by abnormal copper distribution in heart tissue, changes in the biological activity of copper chaperone and copper transporter also promote the occurrence and development of DCM to varying degrees.

The article "The Molecular Mechanisms of Defective Copper Metabolism in Diabetic Cardiomyopathy" was published in 2022. Journal: Oxid Med Cell Longev.

Defective copper metabolism is closely related to a variety of biological processes, such as protein metabolism, lipid peroxidation, and copper metabolism in mitochondria. Copper chaperone is an important carrier of copper input and output in cells and tissues, and its transport obstacle worsens the metabolic disorder and oxidative stress of cuproptosis and accelerates the occurrence and development of cuproptosis. Many studies have shown that pathological changes caused by cuproptosis are mediated by a number of adverse factors. These pathological changes are closely related to the fatal ROS overproduction, changes in copper transporter activity, copper accumulation by glycation induced, and transformation of mitochondrial energy metabolism.

Fortunately, it has been confirmed the effective protective effect of copper ion carrier in the treatment of copper metabolism defects in DCM, such as TETA. Disulfiram can not only target copper ion delivery to cardiomyocytes to improve the copper deficiency in cardiomyocytes but also combine with CP in plasma to reduce the high copper levels in blood to achieve the overall regulation of copper metabolism. What is noticeable is that some copper ion carriers also have the potential role of promoting lipid metabolism, reducing body weight, and treating metabolic diseases, which provides a new treatment direction for DCM in the latest studies.

However, the research on the pathogenesis of defective copper metabolism needs to be further improved, and more measures for different pathways and eight points need to be explored. In addition, many current studies are based on animal or molecular levels, and there are few clinical studies. Therefore, the following problems need to be faced in future research: (1) it is known that glycolysis is inhibited and oxidative phosphorylation is greatly activated in DCM, whether copper supplementation promotes lipid breakdown and exacerbates oxidative stress. (2) Whether we can intervene the regulator FDX1 upstream to achieve the stated goal In protein lipoacylation-mediated cell death，such as killing cancer cells or protecting heart muscle cells. (3) Furthermore, in addition to richer and more mature laboratory studies, more clinical studies should be appropriately carried out.

The article "The Molecular Mechanisms of Defective Copper Metabolism in Diabetic Cardiomyopathy" was published in 2022. Journal: Oxid Med Cell Longev.

## Figures and Tables

**Figure 1:** Metabolic pathway of copper in human body. Transport route of copper in human body: oral intake, in the gastrointestinal tract absorption into the blood, the blood vessels in the copper blue protein combined with albumin and plasma protein transport via portal vein circulation to the liver [26, 30]. After the liver processing, the redistribution to the tissues and organs, such as the skeletal muscle, brain, and heart, widely participates in various life activities [13, 29]. Finally, through metabolism, bile enters the intestine and is excreted in the stool or through the kidney and is excreted in the urine [31, 32]. ATP7A: adenosine triphosphatase 1; CTR1: copper transporter 1; MT: metallothionein (storage of cytosol exceeding copper); SOD1: Cu/Zn superoxide dismutase; GSH: glutathione; CP: ceruloplasmin.

**Figure 2:** Copper ion-mediated cell death in DCM. Copper can mediate various types of cell death in vivo, mainly including apoptosis, autophagy, pyroptosis, and cuproptosis recently discovered via copper-mediated. The different apoptosis pathways are triggered by copper at different time points of the exposure period, as the increase in transcripts was sequential [121]. Apoptosis mainly occurs in mitochondria, nucleus, and endoplasmic reticulum. Autophagy is mainly due to the activation of mTOR-ULK1/2 signaling pathway by copper ion, which is a self-protection mechanism of the body, but excessive autophagy can cause pathological damage to the body [122]. Pyroptosis is caused by copper ion through Fenton/Haber Weiss reactions that occur and involve destructive cell death mediated by ROS [123, 124]. Cuproptosis mainly occurs in cells with high energy demand and abundant mitochondria. Excessive copper ions participate in TCA process under the action of FDX1, which can induce DLAT aggregation and lead to abnormal mitochondrial protein folding, followed by the loss of Fe-S protein, resulting in cell death due to energy metabolism defects [125]. Besides, copper ions can lead to redox imbalance, and the antioxidant defense of GSH and SOD is insufficient to resist the damaging effect of ROS [13].

**Table 1:** Mammalian copper-dependent enzymes.

		Location	Function	Disease consequence	References
CRT1		Plasma membrane and endosomes	High-affinity plasma membrane copper importer; determine the rate of copper import; regulate the REDOX state of Cu^+^	Cardiomyopathy with cardiac hypertrophy and endocardial fibrosis; cardiac hypertrophy	[38, 39]

ATPase	ATP7A	Trans-Golgi network (TGN)	ATP7A: ubiquitously expressed, with the exception of the liver in normal states; regulate the rate of hydrolysis of ATP; regulate copper transport	High frequency of congenital heart disease	[40]
	ATP7B		ATP7B: expressed in the liver and some regions of the brain, placenta, kidney, and mammary tissue; regulate the rate of hydrolysis of ATP; regulate copper transport		

CCS			Copper chaperone for SOD; regulation of SOD1 activity		[41]

CCO		Mitochondria	Electron transfer protein; catalyzes the ultimate step of cellular respiration	Hypertrophic cardiomyopathy, lactic acidosis	[34]

MT		Intracellular	Intracellular copper scavengers; prevention of the deterioration of mitochondrial morphology and reduction in creatine phosphokinase levels; decrease oxidative stress, and apoptosis	Cardiac dysfunction and fibrosis	[42, 43]

SOD	SOD1	Cytosolic	Oxidoreductase; catalyzes the disproportionation of superoxide to molecular oxygen and hydrogen peroxide; restrain oxidative stress, autophagy and apoptosis	Early onset cardiac hypertrophy; cardiac injury (apoptosis and inflammation)	[44]
	SOD2	Mitochondria	The first line of defense against mitochondrial respiration-generated oxidative stress; regulates the activity of SOD1	Lipid peroxidation and activation of apoptosis; myocardial damage; heart failure	[45]
	SOD3	Located extracellularly and expressed in blood vessels	Decreases myocardial apoptosis, fibrosis, and inflammation	Cardiac hypertrophy, left ventricular dilation, fibrosis, IHD, myocardial infarction, and HF	[46–48]

CP		Plasma	An oxidase for NO; converts NO to nitrite in vivo; catalyzes; major Cu carrier in serum; negatively associated with NO	DM, obesity, dyslipidemia, atherosclerosis, IHD, and mortality	[49–52]

LOX		Extracellular matrix	Oxidase; converts lysine into aminoadipic semialdehyde; required for crosslinking of collagen and elastin	Myocardial fibrosis; systolic dysfunction; concentric cardiac hypertrophy	[53, 54]

CTR1: copper transporter 1; ATP7A: copper transporter ATPase 1; ATP7B: copper transporter ATPase 2; CCO: cytochrome c oxidase; ATOX1: antioxidant 1 copper chaperon; MT: metallothionein; SOD: superoxide dismutase; SOD1: Cu Zn superoxide dismutase; SOD2: Mn superoxide dismutase; CP: ceruloplasmin; LOX: Lysyl oxidase.
